# Edible Vitalmelon Fruit Extract Inhibits Adipogenesis and Ameliorates High-Fat Diet-Induced Obesity

**DOI:** 10.1155/2022/2369650

**Published:** 2022-09-22

**Authors:** Lu Guo, Sun Young Park, He Mi Kang, Nam Jun Kang, Dae Youn Hwang, Young-Whan Choi

**Affiliations:** ^1^Department of Horticultural Bioscience, Pusan National University, Miryang 50463, Republic of Korea; ^2^Bio-IT Fusion Technology Research Institute, Pusan National University, Busan 46241, Republic of Korea; ^3^Department of Horticulture, Gyeongsang National University, Jinju 52828, Republic of Korea; ^4^Department of Biomaterials Science, Pusan National University, Miryang 50463, Republic of Korea

## Abstract

Conventional breeding of wild (*Cucumis melo* var. makuwa Makino (CM)) and cultivated (*Cucumis melo* var. reticulatus (CR)) melons is aimed at improving their biological traits. Here, we prepared a nontoxic, bioactive extract of vitalmelon (F1 hybrid) and evaluated its antiadipogenic and antiobesity effects in fully differentiated 3T3-L1 adipocytes and high-fat diet- (HFD-) induced obese C57BL/6 mice. In fully differentiated 3T3-L1 adipocytes, the vitalmelon extract reduced the DMI- (dexamethasone, 3-isobutyl-1-methylxanthine, and insulin-) induced increases in lipid droplet number and intracellular glucose and triglyceride levels. In addition, the extract inhibited 3T3-L1 preadipocyte differentiation by downregulating *PPAR-γ* and target genes *LPL*, *CD36*, *HMGCR*, and *L-FABP*. To investigate the inhibitory effects of the vitalmelon extract on lipid metabolism, we measured serum lipid, hormone, and cytokine concentrations; lipolytic activity; lipid accumulation; and adipogenesis in HFD-fed mice treated with the extract. The HFD+vitalmelon-fed mice showed lower blood cholesterol, free fatty acid, sugar, leptin, and insulin concentrations but higher blood adiponectin concentrations than the HFD-fed mice. Moreover, the HFD+vitalmelon-fed mice showed lower abdominal fat levels, smaller fat cells, lower weight, and fewer lipid droplets in the liver tissue than the HFD-fed mice. Therefore, in HFD-fed mice, vitalmelon regulated lipid metabolism through *PPAR-γ*, highlighting its potential as a promising antiobesity functional food.

## 1. Introduction

Obesity is linked to various diseases, including type 2 diabetes, hypertension, dyslipidemia, fatty liver, gallbladder disease, myocardial infarction, stroke, gout, osteoarthritis, colon cancer, and breast cancer, as well as mental health disorders [1–3]. Obesity is triggered by the disbalance between energy intake and consumption, which results in the growth of adipose tissue due to the promotion of adipogenesis and enlargement of adipocytes [4, 5]. The adipocyte count remains relatively constant throughout adulthood. Recently, long-term high-fat diet (HFD) intake has been shown to preferentially initiate adipogenesis in white adipose tissue, suggesting that fat production is related to obesity and obesity-related chronic diseases. White adipocyte tissue is formed by adipocytes [6–8]. The increase in adipocyte tissue mass *in vivo* is attributed to preadipocyte adipogenesis. Typically, the murine adipocyte cell line 3T3-L1 is used to evaluate adipogenesis and adipocyte differentiation *in vitro*. As such, many studies have investigated the adipogenesis mechanisms and antiobesity effects by inducing the differentiation of 3T3-L1 cells through insulin, dexamethasone, 3-isobutyl-1-methylxanthine, dexamethasone, and rosiglitazone treatment [9–11]. In C57BL/6N mice, HFD administration for 3 weeks increases body weight gain, body fat mass, and liver triacylglycerol levels compared with normal diet administration. Thus, HFD-induced C57BL/6N mice can be used as an animal model of obesity [12, 13].

Adipogenesis is a two-step process in which mesenchymal precursors of the adipocyte system limit the formation of progenitor cells, and the formed progenitor cells differentiate into insulin-sensitive mature adipocytes. At the differentiation stage, preadipocytes undergo early and terminal differentiation through growth arrest, mitotic clonal expansion, and regulation of transcription factors and adipogenesis-related genes, contributing to adipocyte development [14, 15]. Peroxisome proliferator activator receptors (PPARs), including PPAR-*α*, PPAR-*δ*/*β*, and PPAR-*γ*, regulate adipocyte differentiation and lipogenesis. Specifically, PPAR-*γ* controls adipocyte differentiation by regulating lipogenesis-related genes, and PPAR-*γ* ligands have been used in preclinical antiobesity studies. For instance, two PPAR-*γ* antagonists, namely, protopanaxatriol and isorhamnetin, prevent body weight gain in HFD-induced C57BL/6J mice [16, 17]. Furthermore, following isobutyl-methylxanthine, dexamethasone, and insulin (MDI) administration, C/EBP*β* and C/EBP*δ* are expressed first, followed by adipocyte differentiation, which further promotes C/EBP*α* and PPAR-*γ* expression [18, 19].

Wild melons (*Cucumis melo* var. reticulatus (CR)), belonging to the Amber family, are commonly cultivated in Asian countries, including Korea, China, and Japan. It is a net-type melon species characterized by a mesh-like pattern on the rind. It is produced by crossbreeding Ha'Ogen melon, a green-fleshed *cantaloupensis* variety, with Krimka melon, a Russian net-type variety [20–23]. Most CR plant parts, including seeds, roots, bark, leaves, and fruits, are used in herbal medicine owing to their antioxidant, antimicrobial, and anti-inflammatory properties [24–26]. However, these melons are rarely consumed because of their small size and bitter taste. Recently, however, they have been used as breeding materials in Korea because of the characteristic of female flowers set at every node. The “Moneymaker” melon cultivar (*Cucumis melo* var. makuwa Makino (CM)) is an annual creeper of the gourd and cucumber genera, and it is cultivated in many Korean regions. The fruits are cylindrical and oval. Ripe melons vary in color from yellow-green to yellow and have a sweet fragrance and taste [27–33]. CM possesses documented antioxidant, anti-inflammatory, and analgesic properties.

In the present study, we explored the antiadipogenic and antiobesity effects of vitalmelon, the first-generation hybrid of CM and CR melons, on 3T3-L1 cells and HFD-fed mice.

## 2. Materials and Methods

### 2.1. Chemicals

Insulin, rosiglitazone, dexamethasone, HEPES, NaHCO_3_, Oil Red O, sodium deoxycholate, and phenylmethylsulfonyl fluoride were obtained from Sigma-Aldrich (St Louis, MO, USA). SDS, Tween 20, and isopropanol were purchased from GENEray (Shanghai, China). Paraformaldehyde was obtained from TCI (Tokyo, Japan). All antibodies were purchased from Santa Cruz Biotechnology (Dallas, TX, USA). Western blotting loading buffer, Bio-Rad protein assay reagents, and protein markers were obtained from Bio-Rad (Hercules, CA, USA). Triglyceride (TG) and glucose detection kits were purchased from Asan Pharmaceutical (Seoul, Korea).

### 2.2. Breeding Experiment

In May 2018, CM and CR plants were bred following the standard methods in the greenhouse of the Department of Horticulture, Faculty of Agriculture, Gyeongsang National University. Subsequently, CM and CR were crossed. Briefly, seeds of the two varieties were germinated in a horticultural medium (Farm Hannong, Seoul, Korea). Thirty-day-old seedlings of both parents were transplanted into a horticultural mixture in 2,000 mL pots and fertilized every week with a nutrient solution containing macro- and microelements (Mulpure, Daeyu Co. Ltd., Seoul, Korea). Through manually crossbreeding, the female flowers of CR were pollinated with pollen collected from the male flowers of CM. A day before crossing, the female flowers of CR and male flowers of CM were enveloped with butter paper bags. The F1 hybrid produced through the cross between CR and CM parents was designated vitalmelon (*Cucumis melo* var. vitalmelon). Vitalmelon was registered under the accession number KCTC14699BP at the Korean Research Institute of Bioscience and Biotechnology (KRIBB). Plants were crossed in May 2018 and F1 plants were grown in May 2019. Fruits were harvested on days 10, 20, 30, 40, and 50 based on flowering and fruit setting dates.

### 2.3. VW Extract Preparation

Vitalmelons were grown during the late spring of 2019, and the fruits were harvested after 10 days of fruiting development based on the date of anthesis. Freeze-dried vitalmelon fruits were ground to a powder and passed through a 30-mesh sieve. Then, 100 g of the powder was incubated in a water bath with 20-fold volume (*w*/*v*) of distilled water at 80°C for 4 h. Extracts were filtered through Whatman No. 2 filter paper (Whatman International Ltd., Maidstone, England, UK) and then dried using a spray-dryer (Ilshin Lab Co. Ltd., Yangju, Korea) to obtain 60.26 g of VW extract. Spray-dried samples were supplied by Kwangdong Pharm Co. Ltd., Seoul, Republic of Korea. The extract was sealed in a glass bottle and stored at -20°C in a freezer.

### 2.4. High-Performance Liquid Chromatography (HPLC)

HPLC was performed using the Agilent 1100 system (Agilent, Palo Alto, CA, USA) equipped with an injector and dual HPLC pumps. The analysis was performed using the Luna C18 column (4.6 mm × 150 mm inner diameter, 5 *μ*m). The final injection volume was 10 *μ*L. Mobile phases A and B were water and methanol, respectively. The gradient conditions used for the analysis and separation of phenol derivatives were 0 min (30% B) and 0–35 min (30-100%). The flow rate was set to be constant at 0.5 mL min^−1^, and the column temperature was set to 30°C.

### 2.5. Adipocyte Culture and Differentiation

The 3T3-L1 cell line was obtained from the Korea Cell Line Bank (KCLB, Seoul, Korea) and cultured in DMEM containing 10% fetal bovine serum at 37°C in 5% CO_2_ atmosphere. After reaching 80% confluence, the cells were digested and seeded into various culture plates and incubated for 2 days. Untreated 3T3-L1 cells were regarded as the control group, and those treated with 10 *μ*g mL^−1^ insulin (Sigma-Aldrich), 1 *μ*M dexamethasone (Sigma-Aldrich), and 10 *μ*M rosiglitazone (Sigma-Aldrich) (differentiation medium, DMI) were considered the model group. The adipocytes cultured for 2 days were cultured for an additional 2 days in a medium containing insulin. After that, the medium was changed once every 2 days. To evaluate its antiadipogenic effects, VW extract (2, 5, or 10 *μ*g mL^−1^) was treated 2 h before exposure to DMI differentiation medium for 8 days (Figure 1).

### 2.6. Oil Red O Staining

3T3-L1 cells were washed with cold PBS three times, fixed in 4% paraformaldehyde for 0.5 h, and then stained with 0.5% Oil Red O for 30 min. The cells were then washed three times with distilled water to remove excess Oil Red O and observed under a microscope at ×200 magnification (Motic, Xiamen, China). Finally, Oil Red O-positive cells were extracted with isopropanol to quantify intracellular lipid content, and absorbance was measured at 520 nm using the Wallac VICTOR plate reader (Perkin Elmer Corp., Norwalk, CT).

### 2.7. Glucose Uptake Measurement

After inducing 3T3-L1 cell differentiation in 24-well plates using the method described in Section 2.5, the supernatant was harvested on day 8 and centrifuged at 1,000 × *g* for 5 min. To quantify glucose concentration, the collected supernatant (Asan Pharmaceutical, Seoul, Korea) was analyzed using a commercial kit according to the manufacturer's protocol.

### 2.8. TG Measurement

After inducing 3T3-L1 cell differentiation in 24-well plates using the method described in Section 2.5, TGs were extracted using 5% Triton X-100 (Bioshop, Burlington, Ontario, Canada) on day 8. TGs were quantified using a commercial kit (Asan Pharmaceutical, Seoul, Korea) according to the manufacturer's protocol.

### 2.9. Animal Experimental Design

Six-week-old male C57BL/6 mice were obtained from Samtako Bio-Korea Inc. (Osan, Korea). The mice were supplied water and a standard-treated normal diet (10 kcal% fat, Research Diets, New Brunswick, NJ, USA) or an HFD (60 kcal% fat, Research Diets). The animals were maintained at 23 ± 2°C and 50 ± 10% relative humidity under specific pathogen-free conditions and a controlled light cycle (turn on at 08:00 and off at 20:00). All experiments involving C57BL/6 mice were performed at the Animal Resource Center of the Pusan National University Animal Laboratory, which is accredited by the Food and Drug Administration (FDA; Accreditation Unit No. 000231) and AAALAC International (Accreditation Unit No. 001525). The entire animal experimentation protocol was approved by the Pusan National University Animal Ethics Committee (PNU-2020-2709). The mice were randomly divided into five groups (*n* = 10 each): (i) control group: mice receiving a normal low-fat diet; (ii) HFD group: mice receiving HFD; (iii) HFD+HO10 group: mice receiving HFD supplemented with 10 mg kg^−1^ body weight orlistat (Sigma-Aldrich); (iv) HFD+VW01 group: mice receiving HFD supplemented with 5 mg·kg^−1^ VW extract; and (v) HFD+VW25 group: mice receiving HFD supplemented with 25 mg·kg^−1^ VW extract (Table 1). The control diet contained 10 kcal% fat (cat. no. D12450B; Research Diets), and the HFD (cat. no. D12492; Research Diets) contained 60 kcal% fat. The diets were administered for 8 weeks. Food intake and body weight of the mice were measured once every 3 days using an electronic scale (cat. no. AD-2.5; Mettler Toledo, Greifensee, Switzerland) according to the KFDA guidelines. At the end of the experiment, the mice were asphyxiated with CO_2_. Blood samples were collected and used for biochemical analysis.

### 2.10. Serum Biochemical Analyses

Immediately after blood collection, plasma was isolated by centrifuging the tube containing sodium EDTA anticoagulant at 1,500 × *g* for 10 min using a refrigerated centrifuge at 4°C. Plasma, insulin, creatine, leptin, and adiponectin levels were measured using a commercial assay kit according to the manufacturer's instructions. Alkaline phosphatase (ALP), aspartate aminotransferase (AST), alanine aminotransferase (ALT), blood urea nitrogen (BUN), and creatinine (Crea) were measured using an automatic biochemical analyzer (7180 Automatic Analyzer; Hitachi High-Technologies Corp., Tokyo, Japan) from serum.

### 2.11. Hematoxylin and Eosin (H&E) Staining

Fresh adipose and liver tissues were fixed in 4% paraformaldehyde for 24 h, dehydrated using ethanol, and embedded in paraffin. Subsequently, tissues were sectioned at 5 *μ*m thickness, deparaffinized, rehydrated, stained with H&E, and photographed under a microscope.

### 2.12. Protein Extraction and Western Blotting

Proteins from each tissue and cell group were extracted using radioimmunoprecipitation assay (RIPA) lysis buffer containing PMSF. Protein concentration was determined using the Bio-Rad protein assay reagent (Bio-Rad, Hercules, CA, USA). Equal amounts (10 *μ*g) of proteins were separated by SDS–PAGE and transferred to 0.22 *μ*m PVDF membranes (Millipore, Billerica, MA, USA). The membranes were blocked with 5% skim milk buffer for 1 h at room temperature and then incubated with primary antibodies against PPAR-*γ*, LPL, CD36, HMGCR, L-FABP, and *α*-tubulin overnight at 4°C. The membranes were washed three times and incubated with HRP-conjugated goat anti-rabbit secondary antibody for 1 h at room temperature. Protein bands were visualized with an enhanced ECL immunoblotting detection kit and quantified using ImageJ.

### 2.13. Statistical Analysis

All data are expressed as the mean ± standard deviation of at least three independent experiments. Between-group differences were determined using one-way analysis of variance, followed by Duncan's multiple range tests using SPSS 20.0. *P* < 0.05 was considered statistically significant.

## 3. Results

### 3.1. Differences in Fresh Fruit Weight and Cucurbitacin Content between Vitalmelon and Parent Plants

Conventional breeding of CR and CM is aimed at improving their biological traits. Here, we represent the breeding of vitalmelon using efficient, natural, and nontoxic phytochemicals from the extracts of vitalmelon, CR, and CM, such as cucurbitacins A and B. Cucurbitacins are produced by members of the Cucurbitaceae family, such as common squash and gourd, and are the major bioactive compounds produced by this family. Cucurbitacins possess numerous variants, including cucurbitacins A, B, E, and I. Among these, the antiobesity properties of cucurbitacins B, E, and I have been reported. Here, using liquid chromatography with tandem mass spectrometry (LC–MS/MS), we analyzed the concentration of cucurbitacins A and B in freeze-dried samples of vitalmelon fruits and compared the values across harvest times as well as between wild (seed parent: female) and cultivated (pollen parent: male) melons. As shown in Table 2, the cucurbitacin B content of wild melons (seed parent: female) was approximately 40 *μ*g·g^−1^ on a dry weight (DW) basis from fruiting to 10 days postfertilization; this value increased markedly on the 20^th^ day but decreased sharply thereafter. However, in vitalmelon, cucurbitacin B content was very high (50 *μ*g·g^−1^ DW) at the fruiting stage, which slightly decreased (30 *μ*g·g^−1^ DW) at 10 days postfertilization. However, at 50 days postfertilization, the value decreased sharply to trace levels. Cucurbitacin A content showed little change over time.

### 3.2. Effects of VW Extract on 3T3-L1 Adipocyte Differentiation

To investigate their antiadipogenic effects, 3T3-L1 preadipocytes were treated with different concentrations of CR, CM, and VW extracts, followed by DMI induction. Adipogenesis was assessed based on lipid accumulation, as evidenced with Oil Red O staining. All tested extracts suppressed lipid accumulation compared with DMSO. Specifically, 50 *μ*g·mL^−1^ CM extract inhibited lipid accumulation, whereas 1–10 *μ*g·mL^−1^ CR and VW extracts significantly inhibited lipid accumulation. Moreover, VW extract exhibited a stronger inhibitory effect on lipid accumulation than CR extract at concentrations between 1 and 5 *μ*g·mL^−1^. Therefore, VW extract is a more potent antiadipogenic material than CR and CM extracts based on its fruit yield (S1) and adipogenesis inhibitory effects (Figure 2).

### 3.3. Effects of VW Extract on Glucose Uptake and Intracellular TG Accumulation in Fully Differentiated 3T3-L1 Adipocytes

Since glucose uptake and TG accumulation are indicators of fully differentiated adipocytes, we assessed their status in 3T3-L1 adipocytes [34]. DMI increased glucose uptake and TG accumulation, supporting DMI-induced differentiation of 3T3-L1 adipocytes. Conversely, VW extract reduced glucose uptake and TG accumulation in DMI-induced fully differentiated 3T3-L1 adipocytes in a concentration-dependent manner (Figure 3). Thus, VW extract alleviated the DMI-induced differentiation of 3T3-L1 adipocytes by regulating glucose uptake and TG accumulation.

### 3.4. Inhibitory Effects of VW Extract on the Expression of PPAR-*γ* and Its Target Genes in Fully Differentiated 3T3-L1 Adipocytes

The PPAR-*γ* pathway plays a pivotal role in adipocyte differentiation by controlling the transcription of genes involved in lipid transport and accumulation [19, 35]. Therefore, we evaluated the effects of VW extract on the expression of PPAR-*γ* and its target genes. The protein levels of PPAR-*γ* and its target genes, including *LPL*, *CD36*, *HMGCR*, and *L-FABP*, were markedly increased in differentiated adipocytes. However, VW treatment (2–10 *μ*g·mL^−1^) drastically reduced these levels (Figure 4). Thus, VW extract suppressed the protein expression of PPAR-*γ* and its target genes, which are upregulated during adipocyte differentiation.

### 3.5. Inhibitory Effects of VW Extract on Body Weight Gain in HFD-Fed C57BL/6N Mice

We verified the antiobesity effects of VW extract in an HFD-induced C57BL/6N mouse model of obesity. The experiment involved five groups: (i) control group (i.e., mice fed a low-fat diet), (ii) HFD group (i.e., mice fed HFD), (iii) HFD+HO10 group (i.e., mice fed HFD supplemented with 10 mg kg^−1^ body weight orlistat (Sigma-Aldrich)), (iv) HFD+VW01 group (i.e., mice fed HFD supplemented with 5 mg·kg^−1^ VW extract), and (v) HFD+VW25 group (i.e., mice fed HFD supplemented with 25 mg·kg^−1^ VW extract). Initial body weight did not differ among the groups, although mice in the HFD group showed 52.1% body weight gain compared with those in the control group. In the HFD+VW01 and HFD+VW25 groups, body weight gain was inhibited after 8 weeks. At the end of the experiment, body weight of mice in the HFD+VW01 and HFD+VW25 groups decreased by 9.8%, 21.1%, and 22.2%, respectively, compared with that of mice in the HFD group. Moreover, body weight gain in the HFD+VW25 group (0.669 g·day^−1^) was significantly lower than that in the HFD group (0.788 g·day^−1^). Likewise, fat weight in the HFD+VW25 group (2.05 g·day^−1^) was lower than that in the HFD group (3.48 g·day^−1^) (Table 3). Taken together, VW extract reduced weight gain and decreased visceral and subcutaneous adipose tissue mass in HFD-fed mice.

### 3.6. Serum Biochemical Parameters

In previous studies, mice receiving an HFD showed higher AST and ALT levels than those receiving a normal diet. Consistently, in the present experiment, AST and ALT levels in the HFD group were higher than those in the control group, but these levels were reduced following VW extract treatment (Figure 5). Moreover, treatment with VW extract for 10 weeks did not induce liver toxicity. Further, serum lipid levels of C57BL/6 mice fed different diets for 10 weeks were analyzed (Figure 5). Since the increase in subcutaneous visceral fat affects blood TG concentration, fat accumulation in HFD-fed animals increases TG content. Consistently, serum total cholesterol, TG, high-density lipoprotein (HDL), and low-density lipoprotein (LDL) levels were increased in the HFD group compared with those in the control group. Conversely, serum HDL levels were decreased in both HFD+VW01 and HFD+VW25 groups. In addition, serum LDL levels were decreased in the HFD+VW25 group. TG content was increased significantly in the HFD group but only slightly in the HFD+HO10 group, albeit without statistical significance. LDL cholesterol accumulation on arterial blood vessel walls causes arteriosclerosis and heart disease. The risk of disease increases as the blood concentration of LDL cholesterol increases. Meanwhile, HDL cholesterol is considered “good” cholesterol, which removes and transports LDL cholesterol from the blood vessels to the liver. In the present experiment, total cholesterol level was significantly higher in the HFD group than in the control group; however, there were no significant differences among the HFD+HO10, HFD+VW01, and HFD+VW25 groups. Nonetheless, total cholesterol level decreased with increasing VW concentration. LDL cholesterol level in the HFD group was significantly higher than that in the control group but slightly higher than that in the HFD+HO10 group. LDL cholesterol level was decreased in the HFD+VW01 group, albeit without statistical significance, while the value was significantly lower in the HFD+VW25 group than in the HFD group. Blood glucose levels were significantly higher in the HFD group than in the control group, and the value was significantly decreased in the HFD+HO10 group. The VW extract-supplemented diets decreased serum glucose levels, albeit without statistical significance. Blood protein content was significantly increased in the HFD group, and VW extract-supplemented diets significantly suppressed this increase in blood protein content (Figure 5). Overall, the VW extract exhibited antiobesity effects by reducing the blood concentration of free fatty acids and sugar and suppressing the increase in blood cholesterol levels.

### 3.7. Effects of VW Extract on Serum Leptin, Insulin, and Adiponectin Concentration

In a study investigating the association between obesity and insulin concentration, we noted that abdominal fat distribution is closely related to insulin concentration; thus, waist circumference is considered a useful indicator of diabetes induction [11, 13, 36]. In the present study, the increase in insulin concentration in obesity-induced mice (Figure 5) was possibly related to the increase in peripheral abdominal fat due to HFD consumption (Figure 5). As such, serum insulin concentration was augmented in the HFD group (Figure 5) but reduced in the HFD+HO10 group, albeit without statistical significance. Serum leptin and insulin levels were considerably lower in the HFD+VW25 group than in the HFD group (*P* < 0.05). In contrast, serum adiponectin concentration was higher in the HFD+VW01 and HFD+VW25 groups than in the HFD group (Figure 5).

### 3.8. Inhibitory Effects of VW Extract on Liver Lipid Accumulation in HFD-Induced C57BL/6N Mice

The liver is a major organ that produces cholesterol and regulates blood cholesterol levels through lipoprotein synthesis. Live cholesterol concentration is a major indicator of circulatory disease [13]. HFD intake causes fatty liver disease through lipid accumulation [37]. HFD consumption increases lipid accumulation in the liver. In HFD-fed C57BL/6N mice, liver biopsy (H&E staining) was performed following dietary VW treatment for 10 weeks (Figure 6). Lipid accumulation in hepatocytes and differentiation into macrovesicular adipocytes were observed in the HFD group. The number of macrovesicular adipocytes (*P* < 0.001) was significantly reduced in the HFD+HO10 group. The reduction in the number of macrovesicular adipocytes in the HFD+VW01 and HFD+VW25 groups was significant and comparable to that in the positive control (HFD+HO10) group. Therefore, VW extract remarkably improved macrovesicular steatosis (Figure 7).

### 3.9. Effects of VW Extract on Abdominal White Adipocyte Size

HFD-fed mice showed markedly increased epididymal fat mass and enlarged average adipocytes compared with control diet-fed mice (Figure 8). Adipocyte size in the HFD group was approximately 100 *μ*m, being 2.7-fold larger than that in the control group (~37 *μ*m) (*P* < 0.05). In the positive control (HFD+HO10) group, adipocyte size was approximately 50 *μ*m, being two times smaller than that in the HFD group (*P* < 0.05). Compared with that in the HFD group, adipocyte size was significantly reduced in both VW-treated groups in a concentration-dependent manner. Adipocyte size in epididymal adipose tissues was assessed using H&E staining. Adipocyte sizes in the HFD+VW01 and HFD+VW25 groups were significantly decreased to 65 and 60 *μ*m, respectively (Figure 8).

### 3.10. Effects of VW Extract on PPAR-*γ* Signaling

To assess the inhibitory effects of VW on PPAR-*γ* signaling in 3T3-L1 cells, we measured PPAR-*γ* expression level in the liver using western blotting. The expression levels of *PPAR-γ* and its target genes *LPL*, *CD36*, *HMGCR*, and *L-FABP* increased in the HFD group but decreased in the HFD+VW25 group (Figure 9).

## 4. Discussion

Hybridization using pure seedlings is common in plants, and phenotypic changes in hybrid traits have high ecological and evolutionary significance. Crossbreeding also combines desirable traits from both parents to gain the advantages of both and also to express new traits that the parents did not have. Crossbreeding also combines desirable traits from both parents to gain the advantages of both and also to express new traits that the parents did not have. Cucurbitacin is the main bioactive compound produced by members of the Cucurbitaceae family, such as pumpkin and gourd. It has a number of variants including cucurbitacins A, B, E, and I. Cucurbitacins A and B were used as bioactive compounds in CR, CM, and VW to compare and analyze the properties of parental and hybrid species. The present study provides the first direct evidence of the antiobesity effects of vitalmelon, the first-generation hybrid of wild (CM) and cultivated (CR) melons, and offers insights into the regulatory mechanisms underlying these effects in fully differentiated adipocytes and HFD-induced obese mice. Wild and cultivated melons are important horticultural crops belonging to the Cucurbitaceae family. Cucurbitaceous plants find a wide range of applications in food, medicine, cosmetics, perfumery, and culinary fields. Most members of this family possess antioxidant, anti-inflammatory, anticancer, and antibacterial activities. Phytochemically, cucurbitaceous plants contain abundant phenolics, including polyphenols and flavonoids, as well as various other nonphenolic compounds. Among these, cucurbitacins A, B, E, and I are the major compounds in the Cucurbitaceae family. Vitalmelon is the first-generation hybrid obtained by artificially crossing wild melon as the seed parent (female) and cultivated melon as the pollen parent (male). During the flowering period, the cucurbitacin B content of vitalmelon ranges from 30 to 60 *μ*g·g^−1^ DW, although the value decreases over time postharvest.

Obesity results from the abnormal enlargement of subcutaneous fat tissue cells due to the accumulation of excess energy as fat in the body, leading to metabolic disruption because of genetic, endocrine, social, and environmental factors. Therefore, obesity is recognized as an independent disease by itself. According to the World Health Organization (WHO), obesity is a global public health concern that must be addressed [1, 9]. In this context, Cucurbitaceae species have garnered increasing attention worldwide because of their wide spectrum of pharmacological effects, particularly against obesity and its associated disorders [21, 24, 26]. Consistent with this, we observed that vitalmelon alleviated adipogenesis and obesity both *in vitro* and *in vivo*. Specifically, vitalmelon extract regulated adipogenesis and lipid accumulation, which are considered the major drivers of adipocyte differentiation. We further analyzed the antiobesity effects of vitalmelon in an HFD-induced mouse model of obesity using orlistat as the positive control. Regarding weight change in response to diet, a reduction in body weight was observed following the dietary intake of vitalmelon, albeit without statistical significance. In addition, vitalmelon intake reduced visceral adipose tissue mass, adipocyte size, lipid droplet accumulation, and plasma liver enzyme (AST and ALT) and lipid (total cholesterol, HDL cholesterol, LDL cholesterol, and TGs) concentrations in HFD-fed mice. Furthermore, 12 weeks of vitalmelon consumption prevented adverse reactions, such as hepatotoxicity and nephrotoxicity (data not shown). Finally, vitalmelon exerted antiobesity effects by regulating the levels of insulin, adipokines, and leptin, which regulate fat accumulation.

PPAR-*γ*, a ligand-activated transcription factor, is predominantly localized in tissues with active lipid metabolism, including the skeletal muscles, liver, and adipose tissues. Additionally, PPAR-*γ* is expressed in adipose tissues and plays a key role in the molecular mechanisms of adipocyte formation and hyperdifferentiation [19, 35]. Consistently, PPAR-*γ* protein expression level was elevated in fully differentiated 3T3-L1 adipocytes and HFD-induced obese C57BL/6 mice, although this was abrogated by vitalmelon treatment. Next, the expression level of adipocyte fatty acid-binding protein (A-FABP), which plays a pivotal role in regulating fatty acid storage and lipolysis, was significantly increased in fully differentiated 3T3-L1 adipocytes and HFD-induced obese C57BL/6 mice; however, VW treatment significantly inhibited A-FABP expression, exhibiting antiobesity and antiadipogenic effects. Moreover, the expression level of LPL, a major cellular fat transporter protein, increased as a result of TG accumulation in fully differentiated 3T3-L1 adipocytes and HFD-induced obese C57BL/6 mice, and this effect was abolished by VW treatment. Furthermore, CD36, a fatty acid translocase, is a membrane glycoprotein involved in fatty acid absorption. VW treatment markedly attenuated CD36 expression in fully differentiated 3T3-L1 adipocytes and HFD-induced obese C57BL/6 mice. Finally, the expression of HMGCR, a major enzyme in the mevalonate pathway, was markedly suppressed following VW treatment. Therefore, VW exerts antiobesity effects by inhibiting the expression of proteins involved in lipogenesis.

## 5. Conclusions

The present study demonstrated the *in vitro* and *in vivo* antiobesity and antiadipogenic effects of vitalmelon. Specifically, VW extract suppressed obesity by downregulating *PPAR-γ* and its target genes (*LPL*, *CD36*, *HMGCR*, and *L-FABP*), thereby disrupting adipogenesis and lipid accumulation. Our findings highlight the potential of vitalmelon as an antiobesity food.

## Figures and Tables

**Figure 1:** Experimental design of adipocyte differentiation and VW treatment.

**Figure 2:** Aqueous extracts of vitalmelon (VW), *Cucumis melo* var. reticulatus (CR) as seed parent and *Cucumis melo* var. makuwa Makino (CM) as pollen parent, inhibited the differentiation of preadipocytes to adipocytes in 3T3-L1 cells. The cells were induced with DMI or DMI with different concentrations of CR, CM, and VW extracts from days 0 to 8. On the 8^th^ day of differentiation, Oil Red O staining was performed. Optical density (OD) of each sample was measured using an ELISA reader at 520 nm (a). Images were obtained at 200x magnification following Oil Red O staining (b). *n* = 3 for every group, ^∗^*P* < 0.05 and ^∗∗^*P* < 0.01 vs. DMI-differentiated group.

**Figure 3:** Vitalmelon aqueous (VW) extract inhibited (a) glucose uptake and (b) triglyceride (TG) accumulation in 3T3-L1 cells. The cells were induced with DMI or DMI with different concentrations of VW extract from days 0 to 8. On the 8^th^ day of differentiation, the supernatant was collected from each well, and the concentration of glucose and TGs was analyzed. *n* = 3 for every group, ^∗^*P* < 0.05 and ^∗∗^*P* < 0.01 vs. DMI-differentiated group.

**Figure 4:** Vitalmelon aqueous (VW) extract inhibited the expression of PPAR-*γ* and its target genes in 3T3-L1 cells. The cells were induced with DMI or DMI with different concentrations of VW extract from days 0 to 8. On the 8^th^ day of differentiation, total protein was extracted from cells in each group, and the expression of PPAR-*γ* and its target genes was analyzed. *n* = 3 for every group, ^∗^*P* < 0.05 and ^∗∗^*P* < 0.01 vs. DMI-differentiated group.

**Figure 5:** Effects of vitalmelon aqueous (VW) extract on plasma liver enzyme (AST and ALT), lipid (total cholesterol, HDL cholesterol, LDL cholesterol, and triglycerides), total protein, and glucose concentrations in female C57BL/6 mice after 10 weeks. Obesity was induced with a high-fat diet (HFD, 60 kcal%) and different concentrations of VW (1 and 25 mg·kg^−1^ body weight) in C57BL/6 mice. After VW extract treatment for 70 days, the plasma was extracted from the blood of the mice and analyzed. The mice received a normal diet (control), HFD, HFD+10 mg·kg^−1^ body weight orlistat (HO10), HFD+1 mg·kg^−1^ body weight VW extract (VW01), or HFD+25 mg·kg^−1^ body weight VW extract (VW25). *n* = 10 for every group, ^∗^*P* < 0.05 and ^∗∗^*P* < 0.01 vs. HFD group.

**Figure 6:** Serum insulin, leptin, and adiponectin levels in C57BL/6 mice receiving different diets. Obesity was induced with a high-fat diet and different concentrations of VW extract (1 and 25 mg·kg^−1^ BW) in C57BL/6 mice. After treatment with VW extract for 70 days, the plasma was extracted from the blood of the mice and analyzed. The mice received a normal diet (control), HFD, HFD+10 mg·kg^−1^ body weight orlistat (HO10), HFD+1 mg·kg^−1^ body weight VW extract (VW01), or HFD+25 mg·kg^−1^ body weight VW extract (VW25). *n* = 10 for every group, ^∗^*P* < 0.05 and ^∗∗^*P* < 0.01 vs. HFD group.

**Figure 7:** Lipid droplet accumulation in hepatic lobules of C57BL/6N mice receiving different diets. Mice received a control diet (control), a high-fat diet (HFD), HFD+10 mg·kg^−1^ body weight orlistat (HO10), HFD+1 mg·kg^−1^ body weight VW extract (VW01), or HFD+25 mg·kg^−1^ body weight VW extract (VW25). Hematoxylin and eosin were used to stain the liver sections. Magnification = 100x. *n* = 10 for every group, ^∗∗^*P* < 0.01 vs. HFD group.

**Figure 8:** Vitalmelon aqueous (VW) extract decreased the size of abdominal white adipocytes. Visceral abdominal white adipose tissue sections from each group were stained using hematoxylin and eosin. Images were obtained at 100x magnification. Mice received a normal diet (control), a high-fat diet (HFD), HFD+10 mg·kg^−1^ body weight orlistat (HO10), HFD+1 mg·kg^−1^ body weight VW extract (VW01), or HFD+25 mg·kg^−1^ body weight VW extract (VW25). Values are presented as mean ± SEM (*n* = 10). *n* = 10 for every group, ^∗∗^*P* < 0.01 vs. HFD group.

**Figure 9:** Vitalmelon aqueous (VW) extract inhibited the expression of PPAR-*γ* and its target genes in the liver of C57BL/6 mice. Obesity was induced with a high-fat diet (HFD, 60 kcal%) and HFD+25 mg·kg^−1^ body weight VW extract (VW25) in C57BL/6 mice. Following VW extract treatment for 70 days, total protein was extracted from the liver, and the expression of PPAR-*γ* and its target genes was analyzed. *n* = 3 for every group, ^∗^*P* < 0.05 and ^∗∗^*P* < 0.01 vs. HFD group.

**Table 1:** Composition of diets administered in the present study (unit = g%).

	Normal		HFD		HFD+10 mg OT		HFD+1 mg VW extract		HFD+25 mg VW extract	
	10 kcal% fat		60 kcal% fat		60 kcal% fat		60 kcal% fat		60 kcal% fat	
	g%	kcal%	g%	kcal%	g%	kcal%	g%	kcal%	g%	kcal%
Formula										
Protein	19.2	20	26	20	26	20	26	20	26	20
Carbohydrate	67.3	70	26	70	26	70	26	70	26	70
Fat	4.3	19	35	60	35	60	35	60	35	60
Ingredients										
Casein, 30 mesh	200	800	200	800	200	800	200	800	200	800
l-Cystine	3	12	3	12	3	12	3	12	3	12
Corn starch	315	1260	0	0	0	0	0	0	0	0
Maltodextrin 10	35	140	125	500	125	500	125	500	125	500
Sucrose	350	1400	68.8	275	68.8	275	68.8	275	68.8	275
Cellulose, BW200	50	0	50	0	50	0	50	0	50	0
Soybean oil	25	225	25	225	25	225	25	225	25	225
Lard	20	180	245	2205	245	2205	245	2205	245	2205
Mineral mix S10026	10	0	10	0	10	0	10	0	10	0
Dicalcium phosphate	13	0	13	0	13	0	13	0	13	0
Calcium carbonate	5.5	0	5.5	0	5.5	0	5.5	0	5.5	0
Potassium citrate, 1H_2_O	16.5	0	16.5	0	16.5	0	16.5	0	16.5	0
Vitamin mixture V10001	10	40	10	40	10	40	10	40	10	40
Choline bitartrate	2	0	2	0	2	0	2	0	2	0
Orlistat (mg)					10					
Vitalmelon extract (mg)							1		25	
	1,145.8	4,166	860.8	4,207	870.8	4,207	861.8	4,207	885.8	4,207

**Table 2:** Fruit fresh weight and cucurbitacin content at the fruiting stage in seed parent (female), pollen parent (male), and F1 plants^Z)^.

	Sampling days after anthesis					
	0	10	20	30	40	50
Fruit fresh weight (g·fruit^−1^)						
Female	0.4 ± 0.1^bEy)^	3.4 ± 0.8^cD^	5.7 ± 1.1^cCD^	6.4 ± 1.0^cC^	9.5 ± 0.8^aAB^	10.0 ± 1.0^cA^
Male	1.1 ± 0.1^aE^	139.8 ± 4.0^aD^	483.2 ± 22.7^aC^	905.0 ± 142.3^aB^	923.3 ± 109.2^aAB^	1009.7 ± 85.0^aA^
F1	0.5 ± 0.1^bE^	39.1 ± 7.1^bD^	107.7 ± 6.6^bC^	156.2 ± 14.9^bA^	153.8 ± 16.6^bAB^	154.2 ± 15.7^bAB^
Cucurbitacin A (*μ*g·g^−1^ dry weight)						
Female	0.6 ± 0.3^bC^	2.5 ± 1.2^nsB^	3.4 ± 0.9^nsA^	2.9 ± 1.1^aAB^	2.7 ± 0.8^aAB^	1.2 ± 0.5^aBC^
Male	ND	ND	ND	ND	ND	ND
F1	1.5 ± 0.2^aAB^	2.0 ± 0.3^nsA^	2.0 ± 0.5^nsA^	0.7 ± 0.1^bB^	0.2 ± 0.1^bC^	ND
Cucurbitacin B (*μ*g·g^−1^ dry weight)						
Female	45.3 ± 6.1^nsB^	47.5 ± 4.4^aAB^	68.2 ± 11.3^aA^	38.3 ± 9.7^aC^	28.6 ± 4.0^aDE^	22.2 ± 4.5^aE^
Male	ND	ND	ND	ND	ND	ND
F1	55.6 ± 7.2^nsA^	34.1 ± 8.4^bB^	14.1 ± 2.6^bC^	7.5 ± 2.2^bD^	2.5 ± 0.5^bE^	0.4 ± 0.1^bF^

^z)^Wild melon (*Cucumis melo* var. reticulatus (CR)) was crossed with the Moneymaker cultivar (*Cucumis melo* var. makuwa Makino (CM)). ^y)^Values in a column followed by the same lowercase and uppercase letters are not significantly different (*P* < 0.05). Values are presented as mean ± standard deviation (SD) from the analysis of six randomly selected fruits of each variety.

**Table 3:** Body weight and food intake of C57BL/6N mice receiving a high-fat diet for 10 weeks.

Group	Control	HFD	HO10	VW01	VW25
Initial body weight (g)	17.07 ± 0.29	17.03 ± 0.37	16.93 ± 0.41	16.74 ± 0.35	16.34 ± 0.49
Final body weight (g)	23.4 ± 0.6	35.6 ± 1.8	28.2 ± 1.7^∗∗^	32.1 ± 1.6^∗^	28.1 ± 2.0^∗∗^
Body weight gain (g·day^−1^)	0.27 ± 0.021	0.78 ± 0.064	0.49 ± 0.05^∗∗^	0.66 ± 0.05	0.51 ± 0.06^∗∗^
Food intake (g·day^−1^)	2.15 ± 0.21	2.30 ± 0.19	2.19 ± 0.09	1.97 ± 0.05^∗^	1.87 ± 0.13^∗^
Food efficiency ratio (%)	13.0 ± 1.3	34.4 ± 2.8	22.5 ± 0.9^∗∗^	33.9 ± 0.8	27.5 ± 1.8^∗∗^
Liver weight (g·mouse^−1^)	0.85 ± 0.05	0.92 ± 0.04	0.94 ± 0.04	0.87 ± 0.02	0.86 ± 0.04
Kidney weight (g·mouse^−1^)	0.23 ± 0.01	0.26 ± 0.01	0.26 ± 0.01	0.26 ± 0.01	0.25 ± 0.01
Fat weight (g·mouse^−1^)	0.66 ± 0.08	3.48 ± 0.38	1.68 ± 0.33^∗∗^	2.64 ± 0.30^∗^	2.05 ± 0.41^∗^

Mice were fed a control diet (control, 10 kcal% fat), a high-fat diet (HFD), HFD+10 mg·kg^−1^ body weight orlistat (HO10), HFD+1 mg·kg^−1^ body weight vitalmelon aqueous extract (VW01), or HFD+25 mg·kg^−1^ body weight VW extract (VW25). All experimental diets were supplied by mixing with HFD samples. Feed conversion efficiency (%) = [total weight gain/total food intake] × 100. *n* = 10 for every group, ^∗^*P* < 0.05 and ^∗∗^*P* < 0.01 vs. HFD group. Fat weight in epididymal, retroperitoneal, and mesenteric fat.

## Data Availability

The data presented in this study are available on request from the corresponding author.
